The article "Recombinant human klotho protects against hydrogen peroxide-mediated injury in human retinal pigment epithelial cells via the PI3K/Akt-Nrf2/HO-1 signaling pathway" was retracted in 2026. Reasons: concerns about the data; concerns about the results or conclusions.

# Recombinant human klotho protects against hydrogen peroxide-mediated injury in human retinal pigment epithelial cells via the PI3K/Akt-Nrf2/HO-1 signaling pathway

**DOI:** 10.1080/21655979.2022.2071023

**Published:** 2022-05-11

**Authors:** Xuewei Wen, Song Li, Yanfei Zhang, Liang Zhu, Xiaoting Xi, Shuyuan Zhang, Yan Li

**Affiliations:** a Department of Ophthalmology, The First Affiliated Hospital of Kunming Medical University, Kunming, Yunnan, China; b Department of Sport Medicine, The First Affiliated Hospital of Kunming Medical University, Kunming, Yunnan, China

**Keywords:** Klotho, oxidative stress, PI3K/akt-nrf2/HO-1 signaling pathway, apoptosis

## Abstract

Globally, age-related macular degeneration (AMD) is a common irreversible ophthalmopathy. Oxidative stress of retinal pigment epithelial cells is involved in AMD occurrence and development. Klotho is an anti-aging protein with antioxidant properties. We investigated the protective properties of Klotho on hydrogen peroxide (H_2_O_2_)-induced injury of retinal pigment epithelial cells (ARPE-19 cells) and its associated pathomechanisms. We found that Klotho pretreatment for 24 h could up-regulate Bcl-2 levels, decrease the cleaved-caspase-3 and Bax levels, inhibit H_2_O_2_-induced ARPE-19 cell apoptosis, and promote cell proliferation. Klotho pretreatment inhibited the H_2_O_2_-mediated elevations of reactive oxygen species (ROS) in ARPE-19 cells. It enhanced antioxidant activities of the cells and restored the glutathione peroxidase (GPX), superoxide dismutase (SOD2), catalase (CAT), as well as malondialdehyde (MDA) levels to close to the normal level. N-acetylcysteine (NAC), a reactive oxygen scavenger, could reverse the harmful effects of H_2_O_2_ on proliferation, apoptosis, and oxidative stress of ARPE-19 cells. Further, Klotho pretreatment enhanced Akt phosphorylation and expression as well as nuclear translocation of Nrf2 in H_2_O_2_-treated ARPE-19 cells. This indicates that Klotho protects cells from oxidative stress by activating phosphatidylinositol 3 kinase (PI3K)/protein kinase B (Akt)-nuclear factor E2-related factor 2 (Nrf2)/heme oxygenase 1 (HO-1) signaling pathway. Klotho is, therefore, a potential preventive or treatment option for AMD.

## Highlights

- Klotho alleviated injury in H2O2-treated ARPE-19 cells.
- Klotho alleviated oxidative stress and apoptosis of H2O2-treated ARPE-19 cells.
- Klotho activated the PI3K/Akt-Nrf2/HO-1 signaling pathway.
- Klotho alleviated ARPE-19 cell injury by activating the PI3K/Akt-Nrf2/HO-1 signaling pathway.

## 1 Introduction

Globally, AMD is among the major causes of blindness, mainly affecting people aged over 60, resulting in irreversible central vision loss [1]. Due to accelerated metabolism and high oxygen consumption, macula is in a state of physiological oxidative stress [2]. Therefore, retinal degeneration begins in the macula and expands over time [1]. Currently, the exact pathomechanisms of AMD are not completely clear. In the past, AMD was considered to be a disease caused by aging, smoking, high-fat diet, light, alcohol consumption, and other factors [3]. Oxidative stress is considered to be the driving force of all these risk factors [4]. According to the presence or absence of choroidal neovascularization (CNV), AMD occurs into 2 forms: dry (atrophic) AMD and wet (exudative) AMD. According to the clinical signs, AMD is divided into early or late (dry or wet) pathological stages. Early AMD is characterized by the formation of subretinal vitreous membrane warts in the macular region, and its size increases gradually with the passage of time [1]. With the progress of the disease and the accumulation of toxic metabolites, it eventually developed into late AMD, namely wet and dry AMD. In other words, these two kinds of AMD can occur in the same patient at the same time [5]. About 90% of all AMD patients have dry AMD [6], with wet AMD accounting for only 10%. But it progresses rapidly, severe visual impairment can be caused by rupture and bleeding from neovascularization. Vascular endothelial growth factor (VEGF) is considered the most vital pathogenic factor of wet AMD because it can directly lead to the formation of CNV. At present, intravitreal injection of anti-VEGF monoclonal antibody has achieved remarkable results in wet AMD treatment [7]. However, efficacious therapies to prevent the progression of dry AMD are lacking. In addition, some researchers have found that repeated intravitreal injection of anti-VEGF drugs can lead to pathological changes similar to atrophic AMD [8,9], such as choroidal degeneration and endothelial cell loss. Therefore, we still need to find a more effective and safe treatment for both dry and wet AMD.

The article "Recombinant human klotho protects against hydrogen peroxide-mediated injury in human retinal pigment epithelial cells via the PI3K/Akt-Nrf2/HO-1 signaling pathway" was retracted in 2026. Reasons: concerns about the data; concerns about the results or conclusions.

AMD mainly results from oxidative stress occurring in retinal pigment epithelial cells [10]. Thus, modulating oxidative stress in RPE cells may effectively slow down or reverse AMD [11,12]. ROS are essential regulators of signal transduction, gene expression as well as proliferation, migration, and differentiation of cells. However, excessive ROS damages cells and disrupt cell systems [13]. Antioxidant enzymes, such as GPX, SOD2, and CAT, can effectively neutralize ROS, reducing the associated damages [14]. Meanwhile, malondialdehyde (MDA) is a marker for lipid peroxidation and oxidative damage [15]. Researches have shown that natural antioxidants improve eye health and reduce the risk of developing chronic eye diseases, including AMD and cataracts [16,17].

Klotho is an anti-aging protein with numerous health benefits in animals, which translate in to longer lifespan [18]. Overexpression of Klotho slowed down aging and increased lifespan of mice. Intriguingly, inhibiting Klotho accelerated the development of age-related diseases including atherosclerosis, osteoporosis, infertility, and cognitive decline [18]. Klotho can enhance resistance to oxidative stress and inflammation [19–22]. The protein is mainly expressed in the kidney and brain [23] but can also exist as a soluble protein in cerebrospinal fluid, urine, and blood, in exfoliated form [24]. Studies have shown that the Klotho gene family, including α-, β- and γ-Klotho, has been found to be expressed in the human retina, optic nerve, and lens. However, β-Klotho gene was only expressed in the retina and optic nerve [25]. It is reported that Klotho can markedly elevate SOD and GSH-PX activities as well as reduce MDA and lipid peroxidation levels in Human Umbilical Vein Endothelial Cells (HUVECs) [26], and increase the activities of superoxide SOD2 and CAT in mouse tubular epithelial cells (TCMK-1) induced by H_2_O_2_ [27]. Klotho regulates the differentiation and apoptosis of eye lens epithelial cells [28]. Also, researchers have demonstrated marked differences in levels of Klotho mRNA and corresponding proteins between patients with clear lens and those with age-related cataract [25]. In addition, Klotho gene can influence retinal health [29,30]. When RPE cells are damaged, the phagocytic function of POS decreases and the intracellular organelles are damaged, which leads to the formation and accumulation of lipofuscin. Lipofuscin induces photosensitization of RPE cells and further aggravates oxidative stress load and cell damage. In addition, lipofuscin is also associated with cell senescence [10], autophagy [11,31] and angiogenic signals. In one study, it was found that Klotho increased the phagocytosis of primary cultured RPE cells by inducing the expression of MERTK/Ax1/Tyro3 gene [32]. However, it is not clear whether Klotho can protect RPE cells against damage caused by H_2_O_2_.

We assessed the effects of Klotho on H_2_O_2_-induced oxidative stress and retinal pigment epithelial cell apoptosis. Moreover, the regulatory effects of Klotho on PI3K/Akt-Nrf2/HO-1 signaling pathway were investigated.

## 2 Materials and methods

### 2.1 Cell cultures and Klotho pretreatment

Human ARPE-19 cells were obtained from the American Type Culture Collection (Manassas, VA, USA) and passaged in RPMI-1640 medium (Gibco, USA) enriched with 10% (v/v) FBS (Gibco, USA), 100 U/ml of Penicillin, and 100 μg/mL of streptomycin (both from Hyclone, Logan, UT, USA). Incubation was performed at 37°C under 5% CO_2_. Cells in the 3rd–4th passage cells were used in the subsequent experiment. Briefly, the ARPE 19 cells (1 × 10^4^ cells/well) were seeded into 96-well plates and incubated for 24 h with varying doses (20, 50, 100, 200 ng/ml) of recombinant human Klotho protein (aa 34–981, R&D Systems, USA). Cells were treated with varying H_2_O_2_ doses (0–500 μM) for 24 h, to determine the optimal lethal H_2_O_2_ concentration. H_2_O_2_ at the concentration of 300 μM could reduce ARPE-19 cell viabilities to about 50% of that of the control group, and Klotho dose-dependently protected ARPE-19 cells from damage. Therefore, the modeling dose of Klotho (100 ng/ml) and H_2_O_2_ (300 μM) were used in subsequent experiment, the experimental group was divided into Control group, Klotho group, H_2_O_2_ group, Klotho + H_2_O_2_ group, Klotho + H_2_O_2_ + LY294002 group, Klotho + H_2_O_2_ + si-NC, Klotho + H_2_O_2_ + siRNA Nrf2 group, NAC + H_2_O_2_ group. Before treated with H_2_O_2_, the cells were pre-exposed to Klotho (100 ng/ml) for 24 h, PI3K inhibitor (LY294002) (15 μM) (Sigma-Aldrich, USA) for 1 h, Nrf2 siRNA (100 µM) for 12 h or NAC (1 mM and 2 mM) (BestBio, China) for 1 h, respectively. Various assays were performed to evaluate whether Klotho can suppress against H_2_O_2_-induced cell damage.

The article "Recombinant human klotho protects against hydrogen peroxide-mediated injury in human retinal pigment epithelial cells via the PI3K/Akt-Nrf2/HO-1 signaling pathway" was retracted in 2026. Reasons: concerns about the data; concerns about the results or conclusions.

### 2.2 Cytotoxicity analysis

Protective effects of Klotho on H_2_O_2_-mediated ARPE-19 cell damage induced by was assessed using CCK-8 assay. Here, ARPE-19 cells (1 × 10^4^ cells/well) were pretreated with Klotho (20, 50, 100, 200 ng/ml) for 24 h followed by incubation with H_2_O_2_ (300 μM) for 24 h. The culture supernatant was sucked out before adding mixed CCK-8 reagent (10 μl CCK-8 reagent + 100 μl RPMI-1640 medium). Incubation of cells for 2 h was done at 37°C. Optical density (OD) was spectrophotometrically measured at 450 nm. The following formula was employed to calculate cell viability (%): [(experimental group OD – blank group OD)/(control group OD – blank group OD)] × 100.

### 2.3 Real-time quantitative PCR

Total RNA of ARPE-19 cells were isolated by the TRIzol reagent (Invitrogen, USA). The Revert Aid First Strand cDNA Synthesis kit (Thermo Fisher Scientific, Waltham, MA, USA) was used for cDNA synthesis from the RNA. Using Fast-Start Universal SYBR Green Master Mix with ROX (Roche, Basel, Switzerland) and 7500 Real-Time PCR system (Applied Biosystems, Foster City, CA, USA) for 40 cycles to complete amplification. GAPDH was the reference gene. Relative mRNA expressions were determined using the threshold cycles (CTs) normalized. The primer sequences of GAPDH, GPX, CAT, SOD2, α-, β-, and γ-Klotho were presented in Table 1.

The article "Recombinant human klotho protects against hydrogen peroxide-mediated injury in human retinal pigment epithelial cells via the PI3K/Akt-Nrf2/HO-1 signaling pathway" was retracted in 2026. Reasons: concerns about the data; concerns about the results or conclusions.

**Table 1.** Primers used for the evaluation of gene expression

Genes	Forward	Reverse	Product Length
SOD2	GGACAAACCTCAGCCCTAAC	TCAAAGGAACCAAAGTCACG	82
(NM_001322819.2)			
GPX	CATTCGGTCTGGTCATTCTGG	TGGTCGGACATACTTGAGGGT	101
(NM_001329790.2)			
CAT	TTGAAGATGCGGCGAGAC	CCTGTGGCAATGGCGTTA	76
(NM_001752.4)			
klotho-α	TTTGCTTCTATTATTTCTCTCTCCC	ATTTGTAACTTCTTCTGCCTTTCTT	67
(NM-004795.4)			
klotho-β	GAGAAGCATGAGATGAGAGGCAC	TCCAAAAGAAAAGGCAAAGAAAT	51
(NM-175737.4)			
klotho-γ	CACTACCGATTCTCCCTGTCTTG	ATTCCCTTCTTGTTCACCTGCTC	77
(NM-207338.4)			
GAPDH	CGCTGAGTACGTCGTGGAGTC	GCTGATGATCTTGAGGCTGTTGTC	172
(NM_001357943.2)			

### 2.4 Western blotting

ARPE-19 cells were washed thrice in ice-cold PBS before lysis in an ice-cold RIPA lysis buffer with a protease inhibitor (Solarbio, China) for 30 min. Total proteins were extracted from pellets recovered after centrifugation of the lysate at 12,000 × g for 20 min at 4°C. The cytoplasmic and nuclear Nrf2 proteins in ARPE-19 cells were isolated using the nuclear and cytoplasmic proteins extraction kit (Beyotime, China). Quantification of extracted proteins was done by the BCA protein assay kit (Solarbio, China), following the manufacturers’ instructions. Separation of proteins was done on 10% and 12% SDS-PAGE gel, transferred to a PVDF membrane, which was and blocked at room temperature (RT) using 5% skim milk for 2 h. Overnight incubation of the membrane was done at 4°C with primary antibodies, washed thrice using PBS and re-incubated for 2 h at RT with secondary antibodies. The primary antibodies included anti Bax (1:1000, 50,599-2-lg, proteintech, USA), Bcl-2 (1:1000, 12,789-2-AP, proteintech, USA), cleaved-caspase-3 (1:1000, #9662, Cell Signaling Technology, USA), Akt (1:1000, #4685, Cell Signaling Technology, USA), p-Akt (1:1000, #4060, Cell Signaling Technology, USA), Nrf2 (1:1000, NBP1-32,822, Novus Biologics, USA), HO-1 (1:1000, #26,416, Cell Signaling Technology, USA), β-actin (1:1000, #4970, Cell Signaling Technology, USA), GAPDH (1:1000, #5174, Cell Signaling Technology, USA), and anti-histone H3 (1:1000, #4909, Cell Signaling Technology, USA), whereas the secondary antibodies included HRP-conjugated anti-rabbit (1:3000, S0001, Affinity, China) and anti-mouse antibodies (1:3000, S0002, Affinity, China). The proteins bands were detected by enhanced chemiluminescence (ECL) and assessed using Image J software.

### 2.5 Intracellular ROS production

ARPE-19 cells (3 × 10^5^ cells/well) were incubated in 6-well plates with 100 ng/ml of Klotho for 24 h. Cell incubation at 37°C for 20 min was done in serum-free medium supplemented with 10 μM DCFH-DA (Beyotime, China), washed three times using serum-free medium before treatment with H_2_O_2_. The fluorescence intensity was observed using a fluorescence microscope. All ROS levels are shown as a % of normalized levels of the control group (100%).

The article "Recombinant human klotho protects against hydrogen peroxide-mediated injury in human retinal pigment epithelial cells via the PI3K/Akt-Nrf2/HO-1 signaling pathway" was retracted in 2026. Reasons: concerns about the data; concerns about the results or conclusions.

### 2.6 siRNA interference

ARPE-19 cells (2 × 10^5^ cells/well) were inoculated in 6-well plates for 24 h. After transfections with Nrf2 siRNA (100 µM) using lipofectamine 2000 (Thermo Fisher Scientific, USA) for 12 h, the cells were then pre-incubated with Klotho for 24 h prior to H_2_O_2_ treatment. Cytoprotective effects of Klotho were assessed using Western blot or CCK-8 assay.

### 2.7 5-ethynyl-2′-deoxyuridine (EdU) incorporation assay

ARPE-19 cells (3 × 10^5^ cells/well) were inoculated in 6-well plates and accordingly treated before further incubation for 2 h with 37°C preheated EdU (Beyotime, China) working solution (10 µM) at 37°C. Cells were fixed for 15 min in paraformaldehyde (4%) and thereafter incubated at RT for 30 min in darkness, with Click reaction solution. Cell nuclei were then observed by fluorescence microscopy after staining with Hoechst33342 solution.

### 2.8 Immunofluorescence staining

ARPE-19 cells (5 × 10^4^ cells/well) were cultured in 24-well plates with the cell climbing tablets, and after the corresponding treatment, they were fixed in paraformaldehyde (4%) at RT for 15 min, rinsed thrice using PBS, permeabilized for 15 min using 0.3% PBST (Triton X-100) and rinsed twice using 0.1% PBST. Thereafter, 10% goat serum solution was added and incubated at RT for 2 h. Cells were cultured overnight at 4°C in the presence of anti-Nrf2 antibodies (1:200, Novus Biologics, USA), rinsed 3 times using 0.1% PBST before second 2 h incubation with fluorescent secondary antibodies. After rinsing three times using 0.1% PBST, the climbing slides were removed, the cells were fixed on the glass slides with the sealing solution supplemented with DAPI and observed under the fluorescence microscope.

### 2.9 Mitochondrial membrane potential (MMP) assay

ARPE-19 cells (3 × 10^5^ cells/well) inoculated in 6-well plates were treated accordingly. After incubation, they were washed once using PBS buffer, mitochondrial membrane potential measurements were performed by a corresponding detection kit (JC-1) (Beyotime, China). Briefly, the JC-1 working solution was incubated at 37°C in each well for 20 min. Thereafter, we discarded the supernatant and washed the cells twice using JC-1 buffer (1x). The ratio and intensities of red to green fluorescence were detected by fluorescence microscopy and fluorescent enzyme labeling instrument to evaluate MMP.

The article "Recombinant human klotho protects against hydrogen peroxide-mediated injury in human retinal pigment epithelial cells via the PI3K/Akt-Nrf2/HO-1 signaling pathway" was retracted in 2026. Reasons: concerns about the data; concerns about the results or conclusions.

### 2.10 TUNEL assay

The protective effect of Klotho against cell apoptosis was assessed using the TUNEL assay kit (Beyotime, China), as instructed by the manufacturers. Briefly, the cells were treated with Klotho and H_2_O_2_, rinsed once using cold PBS buffer and fixed in paraformaldehyde (4%) for 30 min. Cells were washed once at RT for 5 min in PBS with 0.3% Triton X-100 and rinsed twice using PBS. Thereafter, the 50 μl TUNEL detection solution was supplemented to every well followed by 1 h of incubation at 37°C in darkness. Cells were rinsed thrice using PBS and stained using 100 μl DAPI (1 μg/ml) before observation under fluorescence microscope.

### 2.11 Flow cytometry

The protective effect of Klotho against cell apoptosis was assessed using the Annexin V-FITC/Propidium Iodide (PI) Apoptosis Detection Kit (BD Biosciences, USA). Cells were treated with Klotho and H_2_O_2_, rinsed once using PBS buffer, collected, and centrifuged for 5 min at 1000 rpm. After being washed thrice in PBS, cells (1 × 10^6^ cells/ml) were re-suspended in 1× binding buffer, gently mixed with 5 μl Annexin V-FITC, after which 10 μl Propidium Iodide (PI) staining solution was supplemented to the cells at RT for 10 min in darkness. Annexin V positive cells were noted as apoptotic cells. Apoptotic cell % in each group was evaluated by Flow Cytometry (Thermo Fisher Scientific, MA, USA).

### 2.12 Statistical analysis

Data are shown as mean ± SD and were analyzed by SPSS 18.0 and GraphPad Prism 8.0 softwares. Differences between groups were determined by conducting Student’s t-test. Differences among groups were assessed by ANOVA. P < 0.05 denoted significant outcomes.

## 3 Results

We found that Klotho inhibited oxidative stress as well as apoptosis of H_2_O_2_-treated ARPE-19 cells and increased cell proliferation by regulating the PI3K/Akt-Nrf2/HO-1 pathway. These results provide a new basis for AMD treatment.

### 3.1 Effect of H_2_O_2_ on the level of Klotho in ARPE-19 cells

mRNA levels of α-, β-Klotho in ARPE-19 cells treated with H_2_O_2_ (300 μM) were markedly low, relative to the control group (Figure 1a, b). It is worth noting that differences in expressions of γ-klotho between the H_2_O_2_-treated and control groups were insignificant (Figure 1c).

**Figure 1.** Klotho improved the inhibition H_2_O_2_-induced of ARPE-19 cells proliferation and H_2_O_2_ inhibited Klotho mRNA levels in ARPE-19 cells. (A, B, C) Real-Time qPCR was employed to determine the levels of α-, β- and γ-Klotho mRNA levels of ARPE-19 cells treated with H_2_O_2_ (300 µM) for 24 h. (d) CCK-8 assay was performed to detect the cell viability of ARPE-19 cells induced by H_2_O_2_ with different concentration (0–500 µM) for 24 h, (e) the cytotoxicity of Klotho (20–200 ng/ml) on ARPE-19 cells. ARPE-19 cells were incubated with or without Klotho (20–200 ng/ml) for 24 h then induced by H_2_O_2_ (300 µM) for 24 h. (f) the protective effect of Klotho on H_2_O_2_-induced injury of ARPE-19 cells was performed by CCK-8. ARPE-19 cells were incubated with or without Klotho (100 ng/ml) for 24 h then induced by H_2_O_2_ (300 µM) for 24 h. (g, h) The effect of Klotho pretreatment on the proliferation of H_2_O_2_-induced ARPE-19 cells detected by EdU assay. + indicates with treatment, – indicates without treatment. Each column presented means ± SD (n = 3). *p < 0.05, **p < 0.01, ***p < 0.001, ****p < 0.0001, ‘ns’ represented no statistical significance.

The article "Recombinant human klotho protects against hydrogen peroxide-mediated injury in human retinal pigment epithelial cells via the PI3K/Akt-Nrf2/HO-1 signaling pathway" was retracted in 2026. Reasons: concerns about the data; concerns about the results or conclusions.

### 3.2 Klotho improved the inhibitory effects of H_2_O_2_ on ARPE-19 cell proliferations

The CCK-8 assay revealed that H_2_O_2_ suppressed ARPE-19 cell proliferations by up to 50% after 24 h of incubation (Figure 1d). Further tests revealed that viability levels of cells in Klotho alone and control group were similar (Figure 1e). However, Klotho pretreatment reversed this phenomenon (figure 1f). EdU incorporation assay further validated the inhibitory effects of H_2_O_2_ on proliferation of ARPE-19 cells (decrease in red fluorescence). However, Klotho pretreatment significantly blocked H_2_O_2_-induced damage on ARPE-19 cells (increase in red fluorescence) (Figure 1g, h).

### 3.3 Klotho ameliorated H_2_O_2_-mediated ARPE-19 cell apoptosis

TUNEL assay revealed that Klotho had no effects on ARPE-19 cell apoptosis. Contrarily, compared to control group, H_2_O_2_ treatment significantly triggered apoptosis in ARPE-19 cells. Interestingly, Klotho pretreatment reduced the apoptosis rate from 16.95% to 6.64% (Figure 2a, b), consistent with flow cytometric analyses. Annexin V positive cells (Q2+ Q4) were 20.42% in Klotho pretreatment group compared with 41.23% in H_2_O_2_ group (Figure 2c, d). In addition, the same changes can be observed in mitochondrial membrane potential (MMP) detection. Klotho pretreatment prevented the decrease of MMP H_2_O_2_-treated ARPE-19 cells (Figure 2e, f). Western Blot also indicated that Klotho pretreatment could up-regulate Bcl-2 levels, decrease the cleaved-caspase-3 and Bax levels (Figure 2g, h).

**Figure 2.** Klotho attenuated H_2_O_2_-induced apoptosis of ARPE-19 cells. ARPE-19 cells were incubated with or without Klotho (100 ng/ml) for 24 h then induced by H_2_O_2_ (300 µM) for 24 h. (a, b) The effect of Klotho pretreatment on the apoptosis of H_2_O_2_-induced ARPE-19 cells detected by TUNEL assay; (c, d) Apoptosis ratio was analyzed by being double stained with PI and Annexin V. Annexin V positive cells (Q2+ Q4) was calculated for each group cells. (e, f) fluorescent microscopy images of the mitochondrial membrane potential in ARPE-19 cells with different treatments. JC-1 aggregates show red fluorescence, indicating high mitochondrial membrane potential, and JC-1 monomers show green fluorescence. (g, h) Western Blot was used to determine the expression levels of Bcl-2, cleaved-caspase-3 and Bax in ARPE-19 cells. + indicates with treatment, – indicates without treatment. Each column presented means ± SD (n = 3). *p < 0.05, **p < 0.01, ***p < 0.001, ****p < 0.0001.

The article "Recombinant human klotho protects against hydrogen peroxide-mediated injury in human retinal pigment epithelial cells via the PI3K/Akt-Nrf2/HO-1 signaling pathway" was retracted in 2026. Reasons: concerns about the data; concerns about the results or conclusions.

### 3.4 Klotho attenuated H_2_O_2_-mediated oxidative stress and enhanced the antioxidant capacity of ARPE-19 cells

Intracellular ROS levels in ARPE-19 cells were assessed using DCFH-DA staining. Klotho treatment alone did not alter ROS levels. However, H_2_O_2_ significantly increased ROS as well as MDA levels, and decreased the mRNA levels of GPX, CAT, and SOD2 in ARPE-19 cells. However, Klotho pretreatment decreased the abnormal ROS (Figure 3a, b) as well as MDA (Figure 3c) levels, and modulated the inhibitory effect of H_2_O_2_ against GPX, CAT, and SOD2 in ARPE-19 cells at different degrees, generally close to normal level (Figure 3d-f).

**Figure 3.** Klotho attenuated H_2_O_2_‑induced oxidative stress and lipid peroxidation in ARPE‑19 cells. ARPE-19 cells were incubated with or without Klotho (100 ng/ml) for 24 h then induced by H_2_O_2_ (300 µM) for 24 h. (a, b) Reactive Oxygen Species (ROS) Assay kit was performed to determine ROS levels in ARPE-19 cells. (c) MDA kit was used to detect MDA levels in ARPE-19 cells. (D, E, F) Real-Time qPCR was employed to determine the levels of SOD2, CAT and GPX mRNA levels of ARPE-19 cells. Each column presented means ± SD (n = 3). *p < 0.05, **p < 0.01, ***p < 0.001.

### 3.5 Klotho modulated the effects of H_2_O_2_ in ARPE-19 cells via the PI3K/Akt-Nrf2/HO-1 signaling pathway

H_2_O_2_ treatment elevated p-Akt, Nrf2 (nuclear), HO-1 levels, and decreased Nrf2 (cytosol) levels. However, Klotho pretreatment further increased the expressions of the above proteins (Figure 4a, b). Immunofluorescence staining indicated that Klotho pretreatment markedly increased the nuclear localization of Nrf2 in the cells under oxidative stress (Figure 4c). To determine whether Klotho exerted its effect via the PI3K/Akt signaling pathway, and assess the association between the PI3K/Akt and Nrf2/HO-1 pathways, various assays were performed after treatment with the PI3K inhibitor (LY294002) and siRNA Nrf2. As shown, disrupting the above pathways using LY294002 blocked the cytoprotective effect, including proliferation (Figure 5a-c), apoptosis (Figure 5d, e) and oxidative stress (figure 5f-h) of Klotho on H_2_O_2_-induced injury in ARPE-19 cells, and down-regulated the levels of p-Akt, Nrf2 (cytosol/nuclear), HO-1 proteins (Figure 5k, l). In addition, LY294002 pretreatment induced the decrease of MMP in ARPE-19 cells (Figure 5i, j). This implies that Klotho protects against oxidative stress by initiating the nuclear translocation of Nrf2 and increasing the levels of Nrf2 (cytosol/nuclear), HO-1 proteins via the PI3K/Akt-Nrf2/HO-1 signaling pathway. To validate these findings, we knocked down Nrf2 gene using siRNA. We found this downregulated Nrf2 levels and its downstream HO-1 protein in ARPE-19 cells (Figure 6a, b). Moreover, disrupting of Nrf2 expression also blocked the cytoprotective effect of Klotho against ARPE-19 cells (Figure 6c). Overall, the above findings demonstrated that Klotho confers protection against negative H_2_O_2_-triggered effects on ARPE-19 cells via the PI3K/Akt-Nrf2/HO-1 pathway.

The article "Recombinant human klotho protects against hydrogen peroxide-mediated injury in human retinal pigment epithelial cells via the PI3K/Akt-Nrf2/HO-1 signaling pathway" was retracted in 2026. Reasons: concerns about the data; concerns about the results or conclusions.

**Figure 4.** Klotho modulates the effect of H_2_O_2_ in ARPE-19 cells via the PI3K/Akt-Nrf2/HO-1 Signaling Pathway. ARPE-19 cells were incubated with or without Klotho (100 ng/ml) for 24 h then induced by H_2_O_2_ (300 µM) for 24 h. (a, b) Western Blot was used to determine the expression levels of Akt, p-Akt, Nrf2 (Cytosol/nuclear), HO-1 in ARPE-19 cells. (c) The expression and localization of Nrf2 in ARPE-19 cells was detected by cellular immunofluorescence detection. + indicates with treatment, – indicates without treatment. Each column presented means ± SD (n = 3). *p < 0.05, **p < 0.01, ***p < 0.001.

**Figure 5.** PI3K inhibitor (LY294002) blocked the cytoprotective effect of Klotho on H_2_O_2_-induced injury in ARPE-19 cells. ARPE-19 cells were incubated with Klotho (100 ng/ml) for 24 h, then pretreated with or without LY294002 (15 µM) for 1 h, and then induced by H_2_O_2_ (300 µM) for 24 h. The effect of LY294002 on the proliferation of ARPE-19 cells detected by (a, b) EdU assay and (c) CCK-8 assay. (d, e) The effect of LY294002 on the apoptosis of ARPE-19 cells detected by TUNEL assay; (i, j) fluorescent microscopy images of the mitochondrial membrane potential in ARPE-19 cells with different treatments. JC-1 aggregates show red fluorescence, indicating high mitochondrial membrane potential, and JC-1 monomers show green fluorescence. (f, g) Reactive Oxygen Species (ROS) Assay kit was performed to determine ROS levels in ARPE-19 cells. (h) MDA kit was used to detect MDA levels in ARPE-19 cells. (k, l) Western Blot was used to determine the expression levels of Akt, p-Akt, Nrf2 (Cytosol/nuclear), HO-1 in ARPE-19 cells. + indicates with treatment, – indicates without treatment. Each column presented means ± SD (n = 3). Each column presented means ± SD (n = 3). *p < 0.05, **p < 0.01, ***p < 0.001, ****p < 0.0001.

The article "Recombinant human klotho protects against hydrogen peroxide-mediated injury in human retinal pigment epithelial cells via the PI3K/Akt-Nrf2/HO-1 signaling pathway" was retracted in 2026. Reasons: concerns about the data; concerns about the results or conclusions.

**Figure 6.** Knockdown of Nrf2 blocked the cytoprotective effect of Klotho on H_2_O_2_-induced injury in ARPE-19 cells. ARPE-19 cells were transfected with Nrf2 siRNA (100 µM) using lipofectamine 2000 for 12 h, the cells were then pre-incubated with Klotho for 24 h before H_2_O_2_ treatment. (a, b) Western Blot was used to determine the expression levels of Nrf2, HO-1 in ARPE-19 cells. (c) The effect of siRNA Nrf2 on the proliferation of ARPE-19 cells detected by CCK-8 assay. + indicates with treatment, – indicates without treatment. Each column presented means ± SD (n = 3). Each column presented means ± SD (n = 3). *p < 0.05, **p < 0.01, ***p < 0.001, ****p < 0.0001.

### 3.6 NAC attenuated H_2_O_2_-induced oxidative stress and apoptosis, promoted ARPE-19 cell proliferations

The next experiment explored the potential mechanism of Klotho protecting ARPE-19 cells from injury. CCK-8 found that NAC at 1 mM and 2 mM increased the viabilities and proliferations of cells inhibited by H_2_O_2_ (Supplementary Fig. A, B, C), decreased apoptosis (Supplementary Fig. D, E), and inhibited the increase of ROS (Supplementary Fig. J, K) and MDA (Supplementary Fig. L) levels induced by H_2_O_2_. NAC pretreatment prevented the decrease of MMP H_2_O_2_-treated ARPE-19 cells (Supplementary Fig. F, G). Western Blot also proved that NAC pretreatment inhibited the apoptosis of ARPE-19 cells by up-regulating Bcl-2 levels and decreasing Bax levels (Supplementary Fig. H, I). This protective effect may be achieved by clearing ROS. In addition, H_2_O_2_ treatment suppressed the number of cells and resulted in irregular cell morphology, wrinkling, round, and vacuolar shape, Klotho pretreatment significantly reversed this phenomenon (Supplementary Fig. M).

## 4 Discussion

Clinically, AMD is associated with visual impairment, particularly among the elderly [33]. Meanwhile, AMD mainly results from oxidative stress occurring in retinal pigment epithelial cells [10]. We used H_2_O_2_ to treat ARPE-19 cells to simulate the *in vitro* oxidative stress model of AMD. Hydrogen peroxide mainly caused oxidative damage by causing excessive ROS and attacking antioxidant system, while excessive ROS could induce mitochondrial dysfunction in RPE cells. Mitochondria mainly provide cell energy, maintain signal transduction, and regulate cell cycle. The decrease of cell membrane potential implies dysfunctional mitochondrial, which may lead to cell injury and apoptosis [34]. This is consistent with our research. We found that H_2_O_2_ treatment led to oxidative stress damage in ARPE-19 cells, which inhibited antioxidant enzyme (SOD2, CAT, GPX) levels, induced a large number of ROS and MDA, decreased mitochondrial membrane potential, and finally led to apoptosis. Klotho is an anti-aging protein, which can be divided into membrane type and secretory type. Serum Klotho regulates the function of a variety of hormones, which are mainly involved in calcium and phosphorus metabolism and homeostasis, insulin resistance and ROS production. In a recent study, reduced Klotho levels in aqueous humor in patients with exudative AMD were associated with oxidative stress and inflammation, which supports our finding that H_2_O_2_ treatment inhibited Klotho gene expression in ARPE-19 cells [35]. In addition, pretreatment of ARPE-19 cells with recombinant Klotho protein suppressed ROS and MDA levels induced by H_2_O_2_, elevated antioxidant enzyme (SOD2, CAT, GPX) levels, mitochondrial membrane potential, and inhibited cell apoptosis. Previous reports on Klotho attenuating oxidative stress and apoptosis in cardiomyocytes [36], Periodontal ligament stem cells [37] and lens cells [38] are consistent with our results. It is suggested that Klotho has a protective effect on oxidative stress in ARPE-19 cells.

The article "Recombinant human klotho protects against hydrogen peroxide-mediated injury in human retinal pigment epithelial cells via the PI3K/Akt-Nrf2/HO-1 signaling pathway" was retracted in 2026. Reasons: concerns about the data; concerns about the results or conclusions.

The PI3K/Akt signaling pathway participates in regulation of antioxidant functions in RPE cells [39–41]. and retinal ganglion cells [42]. It is reported that the activation of Akt protects RPE cells from oxidant-mediated cell death under normal conditions and diseases, including AMD [43]. We found that Klotho pretreatment significantly enhanced Akt phosphorylation levels in ARPE-19 cells treated with H_2_O_2_. These findings imply that Klotho can protect ARPE-19 cells from H_2_O_2_-mediated oxidative stress and apoptosis via PI3K/Akt pathway activation. This is in tandem with previous studies, but the difference is that in previous studies, treatment with H_2_O_2_ suppressed the phosphorylation level of Akt, and this difference may be due to different concentrations of H_2_O_2_ (500 μM and 300 μM). Low concentrations of H_2_O_2_ activate Akt signaling pathways to resist oxidative stress damage and prevent apoptosis, but under the action of higher concentrations of H_2_O_2_, the cell self-protection mechanism is decompensated, which is not enough to resist cell injury. Unfortunately, there is no corresponding H_2_O_2_ group (500 μm) in our experiment to verify this conjecture. Nrf2/HO-1 is an antioxidant defense pathway that plays a major role in protecting RPE cells against oxidative damages [44,45]. Mice models revealed that under-expression of Nrf2 can lead to AMD-like pathological changes in the eye [46]. Nuclear factor erythroid 2 related factor 2 (Nrf2) has anti-oxidation effects in mammalian cells [47]. In physiological conditions, Nrf2 binds Kelch-like ECH-associated protein 1 (Keap1) in the cytoplasm [48]. By contrast, conformational changes in the hinge region of Keap1 induced by oxidative stress triggers the release and nuclear transfer of Nrf2. Subsequently, Nrf2 interacts with antioxidant response element (Ares) and activates HO-1, which has been found to effectively block RPE ferroptosis through multiple expression, thus preventing and treating AMD [44]. In this study, we found that H_2_O_2_ treatment could activate the nuclear translocation of Nrf2, while Klotho pretreatment markedly increased the nuclear localization and cytoplasmic expression of Nrf2 in ARPE-19 cells under oxidative stress. This slightly differs from previous reports of Ma *et al*. [28,49] Although both studies have revealed that Klotho can promote nuclear translocation of Nrf2, previous reports have found that Klotho has no effect on the expression of cytoplasmic Nrf2. Some possible reasons for this difference include 1) different cell types (lens cells, cardiomyocytes and retinal pigment epithelial cells used in our study), 2) unique cell culture conditions and unique expression of signal molecules, and 3) different sources of Klotho. In another study, protective effects of Tribulus terrestris in H_2_O_2_-mediated oxidative stress in ARPE-19 cells, H_2_O_2_ of 1 mM suppressed Nrf2 gene and cytoplasmic Nrf2 protein levels, and elevated nuclear Nrf2 protein expressions. Different from our results, tribulus terrestris pretreatment not only promoted the transfer of Nrf2 to the nucleus, but also further decreased the protein expression of cytoplasm. The reason for this difference may be that the concentration of H_2_O_2_ they use (1 mM) is much higher than the concentration we use (300 μM), which leaded to serious oxidative damage to cells. However, Klotho alone has no effect on the expressions of the above proteins, which is similar to previous studies [28], implying that oxidative stress is essential for subsequent Nrf2 nuclear translocation and expression of HO-1 protein. The PI3K inhibitor (LY294002) and Nrf2 knockdown inhibited Nrf2 nuclear translocation and abolished the cytoprotection of Klotho. Overall, Klotho protects against H_2_O_2_-triggered apoptosis and oxidative stress in ARPE-19 cells via the PI3K/Akt-Nrf2/HO-1 signaling pathway. Summarily, for the first time, we demonstrated the beneficial effect of Klotho against H_2_O_2_-stimulated ARPE-19 cell injury. Accordingly, Klotho can be an alternative for early AMD treatment.

The article "Recombinant human klotho protects against hydrogen peroxide-mediated injury in human retinal pigment epithelial cells via the PI3K/Akt-Nrf2/HO-1 signaling pathway" was retracted in 2026. Reasons: concerns about the data; concerns about the results or conclusions.

## 5 Conclusions

In summary, the pretreatment of exogenous Klotho protein suppressed oxidative stress as well as apoptosis of ARPE-19 cells induced by H_2_O_2_, and enhanced the antioxidant activity of ARPE-19 cells. However, PI3K inhibitor (LY294002) and targeted knockdown Nrf2 reversed the cytoprotective effect of Klotho, suggesting that Klotho exerts its cytoprotective effect on ARPE-19 cells via activation of the PI3K/Akt-Nrf2/HO-1 signaling pathway. The present findings reveal new avenues for the prevention and treatment of AMD.

## Supplementary Material

Supplemental Material

## Data Availability

All data generated or analyzed during this study are included in this article.
